# Design of Nonsmooth Groove Tire Bioinspired by Shark-Skin Riblet Structure

**DOI:** 10.1155/2022/6025943

**Published:** 2022-03-27

**Authors:** Congzhen Liu, Hui Meng, Shicheng Lu, Aiqiang Li, Chengwei Xu, Yunfen Sun, Guolin Wang

**Affiliations:** ^1^School of Transportation and Vehicle Engineering, Shandong University of Technology, Zibo 255049, China; ^2^School of Automotive and Traffic Engineering, Jiangsu University, Zhenjiang 212013, China

## Abstract

As one of the major causes of traffic accidents on wet roads, hydroplaning is prone to occur when the traveling speed of a vehicle rises so high that the hydrodynamic pressure between pavement and tires equals inflation pressure. In this condition, the vehicle nearly loses braking and steering capacity. Inspired by the superior drag reduction function of shark-skin riblet, the purpose of this study is to arrange bionic nonsmooth structures at the bottom of longitudinal grooves to promote the hydroplaning performance without affecting other tire performances. A finite element model of 185/60R15 tire was employed and its accuracy was verified by loading tests with CSS-88100 electronic testing instrument. Meanwhile, a fluid domain model was founded by computational fluid dynamics (CFD) method. The simulated critical hydroplaning speed was in accord with that obtained by the NASA empirical formula. Inspired by shark-skin riblet, three kinds of nonsmooth surfaces were exploited. In addition, the drag reduction rate, shear stress, and flow velocity distribution were compared for different grooves. Then, the optimized nonsmooth structure with the best drag reduction effect among three nonsmooth surfaces was arranged at the bottom of longitudinal grooves for bionic tire. Simulation results demonstrated that the bionic tire obviously decreased hydrodynamic lift and increased flow velocities. With these improvements, the critical hydroplaning speed was effectively improved for the bionic tire. These research results can be applied to the promotion of hydroplaning performance without degrading other tire performances.

## 1. Introduction

As the only effective part of vehicles in contact with roads, tires play a key role in supporting loads, cushioning, and force transmission. The grip performance of tires directly affects the safety of vehicles, especially on wet roads. When the driving speed exceeds a certain value on a wet road, the water in the tire contact patch cannot flow out of the tread pattern in time, which will result in hydroplaning [1]. Researches on traffic safety around the world show that tire hydroplaning is one of five major causes of traffic accidents [2]. Therefore, methods to effectively improve hydroplaning performance are attractive in the field of tire research.

Since the 1960s, numerous scholars have conducted in-depth research on tire hydroplaning performance. As for experimental methods, Horne and Joyner from NASA carried out a series of tests to probe the influence of the hydrodynamic pressure, contact area, and inflation pressure on hydroplaning and summarized an empirical formula to predict the critical hydroplaning speed [3]. By testing the pattern groove structure of vehicles on wet roads, Masataka and Toshihiko found the critical hydroplaning velocity increased with the widened pattern groove [4]. Yeager and Tuttle reported an empirical formula to estimate the hydroplaning speed on smooth surface under freely rolling conditions [5]. Through a series of experiments to investigate the influence factors on tire hydroplaning, Gilbert and Robert declared that roove depth, inflation pressure, and ground roughness were positively related to tire hydroplaning performance [6]. In terms of theoretical analysis, Horne et al. derived an expression for predicting the critical hydroplaning speed considering grounding characteristics and inflation pressure [7]. By dividing the contact area on wet roads into three parts, Moore proposed the concept that tire hydroplaning could be divided into dynamic hydroplaning and viscous hydroplaning [8]. According to the energy conservation law to estimate the braking distance of vehicles, Cho et al. presented a braking interval equivalence theory on wet roads [9]. In the context of finite element simulation, Fwa and Ong studied the influence of the spacing, depth, and width of transverse grooves on the critical speed [10, 11]. With simulation analysis to explore the influence of the tread groove on hydroplaning speed, S. Kumar and A. Kumar detected that the critical speed increased by 5.5 km/h and 1.6 km/h for every 1 mm increase in the width and depth of the transverse groove, respectively [12].

In the above studies, experiments, theoretical analysis, and simulations were adopted to investigate the various influencing factors on hydroplaning performance. All offered considerable contributions to hydroplaning improvement. However, the effects of the hydroplaning optimization methods above on other tire performances were scarcely probed. The experimental method is more consistent with the actual hydroplaning phenomenon. Nevertheless, due to the harsh experimental conditions and high costs, the finite element simulation method has become the mainstream approach. Many achievements have been made through the simulation method, but there are still some problems to be solved. For instance, researchers usually deal with the macrostructure of tread pattern to improve the hydroplaning performance. However, a change in the pattern macrostructure may lead to degradation in other performances, such as grip and wear resistance. Therefore, a method that can improve hydroplaning performance without altering the macrostructure of tread groove is pursued.

At present, bionic non-smooth structures have been used in the field of fluid drag reduction [13, 14]. Walsh studied drag reduction on grooved surfaces and found that shark-skin had downstream grooves [15]. Wind tunnel tests showed that the geometry of the grooves had a great influence on drag reduction performance. With wind tunnel tests and oil pipe tests on bionic shark-skin structure, Bechart et al. found that the three-dimensional ribbed surface reduced turbulent shear stress by 7.3% in comparison with smooth surface [16]. Reif found longitudinal microstructural grooves on shark-skin surface could interact with fluid, stabilize the boundary layer and reduce the adhesion resistance of water [17, 18].

In this paper, three bionic nonsmooth structures are designed to improve the critical hydroplaning speed without affecting other tire performances. A finite element model of 185/60R15 tire was established, and the accuracy of the model was verified by comparing the simulation results with test data in static condition. With computational fluid dynamics (CFD) method, a fluid domain model was founded for hydroplaning analysis. Then, the results were compared with NASA empirical formula to verify the rationality of the hydroplaning model. According to boundary layer theory, the simulation structure parameters were determined. Three kinds of nonsmooth surfaces were designed with the inspiration of shark-skin riblet, and the drag reduction mechanism was analyzed. Finally, an optimized nonsmooth structure was placed at the bottom of longitudinal grooves. Simulation results showed that the bionic nonsmooth groove increased the thickness of the boundary layer, improved the mainstream velocity, and reduced the hydrodynamic pressure without transforming the macrostructure of tread groove. With these improvements above, the bionic tire promoted the hydroplaning performance and driving safety on wet roads.

## 2. Model Establishment and Verification

### 2.1. Finite Element Model

The deformation of tread pattern directly affects the hydroplaning performance. In addition, material nonlinearity and geometric nonlinearity of tires increase the model complexity. On the precondition of model accuracy for reliable results, it was necessary to simplify the tire model reasonably. The 185/60R15 tire finite element model with complex tread pattern was composed of tread, sidewall, and rim. In the simulation analysis, the tread and sidewall were defined as homogeneous orthotropic elastic materials. Meanwhile, the road and rim were defined as rigid bodies. Besides, the shell model was adopted for both tire and road surface.  Figure 1 shows the simplified finite element model.

Reasonable boundary conditions are necessary to ensure the accuracy of simulation results. Improper settings result in the simulation failing to converge [19]. To avoid tangential relative sliding or normal separation, a bonded line contact was chosen for the boundary of rim and sidewall. A friction coefficient of 0.70 between the tire and road was selected [20]. Meanwhile, the total time was set to 2 s, and the time step was set to 0.01 s. Inflation pressure was imposed to the inner surface of the tire at 0 ~ 0.20 s with its direction vertical to the inner surface. Then, the load of 4000 N was applied to the outer side of the rim in the interval of 0.20~0.60 s and remained constant after 0.60 s. In this process, the rigid road was subject to fixed constraints.

### 2.2. Hydroplaning Model

Actually, fluid covers the whole surface on wet road. According to the actual rolling of the tire on wet road, the amount of the calculation was huge in simulation analysis, which was difficult to achieve. To improve the computational efficiency during the process of hydroplaning, it was reasonable and acceptable to constrain the direction of the tire along the road and impose a certain speed on the water. In this situation, the water moved relative to the motionless tire. The length, width, and height of the water model were set at 200 mm, 200 mm, and 10 mm, respectively [21]. To obtain the fluid domain, the tire shell model was transformed into solid, then Boolean subtraction was performed on water model. The fluid domain was meshed into independent tetrahedral elements. Accordingly, 364505 cells and 76043 nodes were generated, as shown in Figure 2.

The material property of the fluid domain was set to water. To ensure that no water penetrated inside the tire, boundary conditions were defined in the fluid domain, as expressed in Figure 3. The inlet of the fluid region was set as the velocity inlet, and the water proceeded with an acceleration of 50 m/s^2^. In the simulation process, the time step of the fluid domain calculation should be consistent with the tire static calculation. After the tire was inflated and loaded, the water started from zero and increased to 30 m/s within 0.60~1.20 s. After 1.20 s, the flow velocity remained constant. The outlet and side of the fluid domain were set as pressure outlets, and the hydrostatic pressure relative to the reference pressure point was set to 101.32 kPa [22, 23]. Then, the bottom surface was set as sliding wall without shear force, and its velocity was in accordance with the water velocity. Finally, the contact surface of the fluid domain was defined as the mechanical information transmission surface between the tire and water layer.

In the simulation analysis of tire hydroplaning, isothermal and incompressible viscous fluid model was selected for water. The control equation and turbulence model were N-S equation and Realizable *k*‐*ε*, respectively. Meanwhile, the wall function was defined as the standard wall function. The flow field was initialized by hybrid initialization, and SIMPLEC algorithm was used to obtain the solution of flow field [24, 25].

### 2.3. Model Verification

As for tire hydroplaning, tread deformation is of great significance to drainage. To verify the accuracy and reliability of the finite element model, CSS-88100 electronic testing instrument was used for loading tests, as shown in Figure 4.

The test procedure was as follows. To prevent the influence of temperature on the tire, the indoor ambient temperature was kept at 25°C. Then, the tire was left in this thermostatic room for 72 hours before test. Six sample points were evenly arranged on the sidewall of the tire. The mean value of radial deformation at different positions under a certain load was calculated for accuracy. Furthermore, carbon papers and white papers were placed between the tire and test board to collect the contact patch at different loads. Accordingly, a dedicated computer was used for load control and data storage. For each test, the data were recorded after the load maintaining for 2 min. Finally, the load-deformation curves and contact patches under different loads and inflation pressures were acquired.

Figure 5 shows the comparison of load-deformation curves between test data and simulation results. The tendency of all curves was approximately linear. It was clear that the simulation results were close to the experimental results. Moreover, the maximum distinction was 5.31%, which indicated the high accuracy of the tire finite element model.

Figure 6 and Table 1 express the comparison of tire contact patches under 4 kN with 210 kPa inflation pressure. The profile and pressure distribution are extremely similar. Besides, the maximum relative deviation of contact patch dimensions between the test and simulation was 3.17%. Both the comparisons of load-deformation and contact patch indicated the accuracy and credibility of the finite element model. Similar results can be seen at other loads and inflation pressures. Therefore, the finite element model could be used for further analysis reliably.

Based on numerous hydroplaning tests, the NASA empirical equation was one of the classic equations for predicting critical hydroplaning speed [26]. Its effectiveness has been recognized by many scholars [27]. The empirical equation was

(1) $$\begin{array}{c} V_{h}=6.35\sqrt{P}, \end{array}$$

where *V*_h_ represented the critical hydroplaning speed in km/h and *P* was the inflation pressure in kPa. In the conditions of 210 kPa inflation pressure, 4 kN load, and 10 mm water film, the predicted critical hydroplaning speed was 92.02 km/h according to Eq. (1). Under the same conditions, the simulated hydroplaning speed was 89.10 km/h. The relative deviation between the empirical equation and simulation was 3.27%, which manifested the rationality of the hydroplaning model. Similar approaches were adopted by previous studies [28, 29].

## 3. Drag Reduction of Bionic Nonsmooth Surface

### 3.1. Bionic Nonsmooth Groove

Riblet structures aligned in the flow direction of shark-skin are famous for drag reduction in the turbulent-flow regime [16], as shown in Figure 7. Inspired by the riblet structure characteristics of shark-skin, three kinds of nonsmooth groove structures were designed and arranged at the bottom of tire longitudinal pattern groove along the flow direction, as shown in Figure 8. The length, width, and depth of the computational domain were 30mm, 7mm, and 8mm, respectively, as shown in Figure 8(a). The parameters of the bionic nonsmooth grooves are shown in Figure 8(b), where r represents the radius of the riblet, d represents the interval of bionic groove II, and r_0_ represents the interval arc radius of bionic groove III.

To ensure that the microstructure grooves influence the internal structure of the boundary layer and achieve the effect of drag reduction, the size of the grooves should not be too close to the thickness of the boundary layer [31]. The form of water in the groove was mainly turbulent flow. Thus, the boundary layer thickness could be determined according to the turbulent boundary layer thickness formula:

(2) $$\begin{array}{c} \text{d}=0.381{{xRe}_{x}}^{-\frac{1}{5}}, \end{array}$$

(3) Rex=Vxv,

where *x* was the characteristic length, Re_x_ was the Reynolds number, *V* was the constant velocity, and *v* was the kinematic viscosity. For the maximum boundary layer thickness of the fluid domain calculated was approximately 0.91 mm, the groove radius r was set at 0.40 mm, the interval *d* was 0.20 mm, and the radius of the interval arc r_0_ was 0.10 mm.

### 3.2. Mesh and Boundary Condition of Computational Domain

The triangular prisms and tetrahedron elements were selected for computational domain. Due to the existence of bionic microstructures, it was necessary to adopt refined mesh for the domain near the bionic groove surface [32], as shown in Figure 9. The general grid size of computational domain was approximately 0.30 mm. However, the grid near the bionic structure surface was approximately 0.05 mm. Additionally, the grid in the first layer of the turbulent boundary was 0.01 mm. Within the turbulent boundary, the growth rate and total layers were set at 1.20 and 10, respectively.

The boundary conditions of the computational domain were consistent with the tire hydroplaning model above. The only difference was the entry speed. In the computational domain, six inflow speeds (60 km/h, 70 km/h, 80 km/h, 90 km/h, 100 km/h, and 110 km/h) were defined as the entry boundary conditions.

### 3.3. Model Verification

The incompressible flow state could be described by the Bernoulli equation:

(4) $$\begin{array}{c} Z_{a}+\frac{p_{a}}{\rho g}+\frac{\alpha_{a}{v_{a}}^{2}}{2g}=Z_{b}+\frac{p_{b}}{\rho g}+\frac{\alpha_{b}{v_{b}}^{2}}{2g}+h_{w}, \end{array}$$

where *a*, *b* represented different cross sections within fluid domain, *Z* is the positional potential energy, *p*/*ρg* represented pressure potential energy, *α*_*a*_, *α*_*b*_ were the kinetic energy correction coefficients resulting from frictional resistance and energy loss (The values were equal to 1 when the fluid undergoes turbulent flow and 2 when the fluid undergoes laminar flow), *αv*^2^/2*g* represented the kinetic energy, and *h*_*w*_ was the energy loss of a unit mass fluid flowing between two cross sections.

(5) $$\begin{array}{c} h_{w}=\zeta_{c}\frac{L}{d}\frac{v^{2}}{2g}, \end{array}$$

where *ζ*_*c*_ was the drag coefficient, *L* was the length of the groove, and *d* was the hydraulic diameter of the groove. According to the equations above, the flow quantity of the outlet cross section could be deduced as follows:

(6) $$\begin{array}{c} Q=v_{b}A_{b}=A_{b}\frac{1}{\sqrt{1+\zeta_{c}\left(L/d\right)}}\sqrt{2g\left[\left(\frac{P_{a}-P_{b}}{\rho g}\right)+\frac{v_{a}}{2g}\right]}. \end{array}$$

The drainage capacity of the tread grooves has an important influence on hydroplaning. Generally, higher drainage capacity means smaller fluid resistance and higher hydroplaning speed [33].  Table 2 shows the average flow quantities at the outlet of the smooth groove and bionic grooves with different inflow speeds. Obviously, each outlet flow quantity of the three bionic grooves was bigger than that of smooth groove at different speeds researched, which indicated flow resistance reduction and drainage capacity improvement of bionic nonsmooth grooves. Besides, the flow quantity of groove I was biggest among the three bionic grooves.

High dynamic pressure results in an increase of the flow resistance and energy loss [34].  Table 3 shows the dynamic pressure at the bottom of grooves with different inflow velocities. It can be seen that the dynamic pressure increased with the increase of speed for each groove. At the same speed, the dynamic pressures of the bionic grooves were lower than that of the smooth groove, and the dynamic pressure of groove I was the least. Results above showed that bionic nonsmooth grooves reduced dynamic pressure and flow resistance.

The drag reduction effect of bionic grooves was evaluated by the drag reduction rate *R* and calculated by Eq. (7).

(7) $$\begin{array}{c} R=\frac{\left(\tau_{s}-\tau_{b}\right)}{\tau_{s}}\times 100\%, \end{array}$$

where *τ*_*s*_ was the shear stress of smooth groove, *τ*_*b*_ represented the shear stress of bionic grooves.  Figure 10 describes the drag reduction rates of bionic grooves at different speeds. Each bionic groove exhibited drag reduction effect. At the speed of 90 km/h, bionic grooves displayed the best drag reduction effect among other speeds researched. Moreover, the drag reduction effect of the groove I was better than those of grooves II and III, which was consistent with the results of dynamic pressure.

### 3.4. Drag Reduction Mechanism of Bionic Nonsmooth Structure

Generated by the interaction between the wall and fluid, the shear stress reflected the viscous resistance of the fluid [35].  Figure 11 displays the shear stress nephogram at the speed of 90 km/h. With reference to smooth groove, the shear stress value was almost constant in the whole fluid domain, with only slight increase in the inlet. It was clear that each shear stress of bionic grooves at the inlet was greater than that of the smooth groove. This could be attributed to the concavo-convex surface of the inlet. However, with the continuous inflow of fluid, the shear stress of bionic grooves decreased gradually. Obviously, as for the middle and rear region of fluid domain, the shear stress of the bionic grooves was less than that of the smooth groove. This indicated the reduction of viscous resistance for bionic grooves. Additionally, low shear stress area of the groove I was larger than that of the other two bionic grooves, which signified the best viscosity reduction effect.

Figure 12 exhibits the velocity distributions along vertical (*Y*) direction (Indicated in Figure 11). With the same *Y* values, each speed of bionic grooves was obviously lower than that of the smooth groove. Slow velocity variations meant small velocity gradient, which resulted in small viscous shear stress and Reynolds shear stress. Thus, the bionic grooves realized drag reduction. Moreover, groove I displayed the best drag reduction effect.

## 4. Hydroplaning Performance of Bionic Tire

### 4.1. Tire Hydroplaning Simulation

The comparisons above show that groove I had the best drag reduction effect among three researched bionic structures. Therefore, groove I structure was arranged at the bottom of the tire longitudinal grooves, as shown in Figure 13.

Figure 14 shows the variations of hydrodynamic lift with time. The tire was considered to hydroplaning when the hydrodynamic lift was equal to the load. For both the smooth-groove tire and bionic tire, the loads were applied gradually within 0–0.60 s and kept constant after 0.60 s. The grooves discharged water fast enough for the low speed in 0–0.60 s, and the hydrodynamic lift increased slowly. With the continuous increase of speeds, the water could not be discharged completely. Therefore, the hydrodynamic lift increased rapidly after 0.60 s and reached the maximum after 1.20 s. However, complete hydroplaning happened at 1.09 s for the smooth-groove tire and 1.18 s for the bionic tire. Simulation results showed that the critical hydroplaning speeds of the smooth-groove tire and bionic tire were 89.10 km/h and 97.20 km/h, respectively. This indicated the critical hydroplaning speed of the bionic tire was 9.10% higher than that of the smooth-groove tire.

### 4.2. Flow Field Characteristics of the Bionic Tire

To explore the hydroplaning mechanism of the bionic tire, the hydrodynamic pressure and flow velocity of the fluid domain at 90 km/h were compared for smooth-groove tire and bionic tire.

Figure 15 shows the distributions of hydrodynamic pressure. It was clear that the hydrodynamic pressure mainly distributed at the leading edge, shoulders, and longitudinal grooves. For both tires, the hydrodynamic pressure of two central longitudinal grooves was significantly higher than that of two lateral longitudinal grooves, which indicated that the central longitudinal grooves played the dominant role in drainage. However, the hydrodynamic pressure in the two central longitudinal grooves of the bionic tire was distinctly smaller than that of the smooth-groove tire. A reasonable interpretation was the bionic tire grooves reduced flow resistance and expedited the water drainage. With this improvement, the bionic tire improved hydroplaning performance.

The drainage capacity of tire longitudinal grooves has a significant effect on hydroplaning performance.  Figure 16 exhibits the velocity distributions of longitudinal grooves at different positions. Within 0–5 mm, the flow velocity decreased a little and then sharply increased to a maximum. The possible reason was the pressure differential between the leading edge and the front of longitudinal grooves. After velocity maximums, probably due to the wall resistance and the drainage effect of transverse grooves, the velocity decreased gradually until the end. Moreover, both the flow velocities at central and lateral longitudinal grooves of bionic tire were higher than those of the smooth-groove tire. This could be attributed to the bionic nonsmooth structures. High flow velocity in grooves indicated high critical hydroplaning speed.

## 5. Conclusions

In this paper, to improve the tire hydroplaning performance without affecting other performances, three novel bionic nonsmooth structures are explored with the inspiration of shark-skin riblet. Comparative analyses on the flow quantity, dynamic pressure, and velocity distribution with fluid structure coupling method indicate that groove I exhibits the best drag reduction effect. Therefore, groove I structure is arranged at the bottom of the tire longitudinal grooves along the flow direction. Simulation results about hydrodynamic lift, hydrodynamic pressure, and velocity distributions show that the critical hydroplaning speed of bionic tire is higher than that of smooth-groove tire. Thus, this approach can be applied to the promotion of tire hydroplaning performance on wet roads. It should be noted that the proposed nonsmooth structure only modifies tire longitudinal grooves but not the tread pattern. Other tire properties are considered unaltered. To ensure the service life and safety, it will be worthwhile to comprehensively analyze grip, rolling resistance, and durability, especially noise.

## Figures and Tables

**Figure 1:** Finite element model of tire and road.

**Figure 2:** Fluid domain model and meshing.

**Figure 3:** Boundary conditions of tire hydroplaning model.

**Figure 4:** Static loading test.

**Figure 5:** Load-radial deformation.

**Figure 6:** Comparison of tire contact patches. (a) Simulation result and (b) Test result.

**Figure 7:** Scale patterns of the Galapagos shark [30].

**Figure 8:** Bionic pattern groove model. (a) Calculation domain and (b) three bionic nonsmooth grooves.

**Figure 9:** Mesh of computational domain.

**Figure 10:** Drag reduction rates of bionic grooves.

**Figure 11:** Shear stress comparison. (a) Smooth-groove; (b) Bionic groove I; (c) Bionic groove II; and (d) Bionic groove III.

**Figure 12:** Velocity distributions along longitudinal grooves.

**Figure 13:** The bionic tire model.

**Figure 14:** Hydrodynamic lift.

**Figure 15:** Distributions of hydrodynamic pressure. (a) Smooth-groove tire; (b) Bionic tire.

**Figure 16:** Velocity distributions of longitudinal grooves at different positions. (a) Central longitudinal grooves; (b) Lateral longitudinal grooves.

**Table 1:** The test and simulation results of contact patch dimensions.

Items	Test	Simulation	Relative deviation (%)
Length (mm)	115.90	112.32	3.17
Width (mm)	131.10	127.53	2.64

**Table 2:** Flow quantity of outlet with different inflow speeds.

*V* (km/h)	*Q* (kg/m^2^·s)			
	Smooth-groove	Bionic groove I	Bionic groove II	Bionic groove III
60	17123.6	17705.8	17657.8	17548.2
70	19537.2	20234.7	20179.9	20045.1
80	22465.9	23339.8	23234.2	23079.2
90	25469.2	26490.5	26375.9	26172.1
100	27982.5	29012.3	28917.1	28732.4
110	30422.5	31453.8	31380.8	31192.1

**Table 3:** Dynamic pressure at the bottom of grooves with different inflow speeds.

*V* (km/h)	*P* (kPa)			
	Smooth groove	Bionic groove I	Bionic groove II	Bionic groove III
60	42.74	28.823	29.849	30.077
70	67.882	43.382	43.391	45.056
80	100.133	60.719	62.518	64.037
90	151.364	82.629	83.725	87.038
100	184.789	101.137	113.823	115.121
110	206.368	121.593	135.058	138.584

## Data Availability

The data used to support the findings of this study are available from the corresponding author upon request.
